# Effectiveness of Noninvasive Positive Pressure Ventilation Combined with Enteral Nutrition in the Treatment of Patients with Combined Respiratory Failure after Lung Cancer Surgery and Its Effect on Blood Gas Indexes

**DOI:** 10.1155/2022/1508082

**Published:** 2022-06-29

**Authors:** Yongjun Zhang, Lanbo Liu, Dawei Li, Dongsheng Zhou

**Affiliations:** ^1^Department of Cardiothoracic Surgery, Xiangyang Central Hospital, Affiliated Hospital of Hubei University of Arts and Science, Xiangyang 441021, Hubei, China; ^2^Department of Cardiothoracic Surgery, Xiangyang No. 1 People's Hospital, Hubei University of Medicine, Xiangyang 441000, Hubei, China

## Abstract

**Purpose:**

To investigate the effect of noninvasive positive pressure ventilation (NIPPV) combined with enteral nutrition support in the treatment of patients with combined respiratory failure after lung cancer surgery and its effect on blood gas indexes.

**Methods:**

A total of 82 patients with combined respiratory failure after lung cancer surgery who were treated in our hospital from March 2016∼September 2021 were selected as the research subjects, and according to the random number table method, they were equally divided into the parenteral nutrition group (*n* = 41) with NIPPV + parenteral nutrition support treatment and the enteral nutrition group (*n* = 41) with NIPPV + enteral nutrition support treatment. The curative effects of two groups after treatment were compared, and the pulmonary function indexes (maximum expiratory pressure (PEmax), maximum midexpiratory flow rate (MMF), and maximum ventilation volume (MVV)), blood gas indexes (blood oxygen partial pressure (PaO_2_) and partial pressure of carbon dioxide (PaCO_2_)), oxygen metabolism indicators [mixed venous oxygen tension (PvO_2_) and central venous oxygen saturation (ScvO_2_)], nutritional status indicators (hemoglobin (HGB), serum albumin (ALB), and total protein (TP)), and nutritional score before and after treatment in two groups were detected, and the 6-month follow-up of the two groups was recorded.

**Results:**

After treatment, the total effective rate of the enteral nutrition group 95.12% (39/41) was higher than that of the parenteral nutrition group 80.49% (33/41) (*P* < 0.05). At 3, 12, 24, and 48 hours after the operation, the levels of PEmax, MMF, and MVV in two groups were higher than those before treatment, and the enteral nutrition group was higher than the parenteral nutrition group at the same time point (*P* < 0.05). At 3, 12, 24, and 48 hours after the operation, the PaO_2_ levels in two groups were higher than those before treatment, and the PaCO_2_ levels were lower than those before treatment. The PaO_2_ levels in the enteral nutrition group were higher than those in the parenteral nutrition group at the same time point, and the PaCO_2_ levels were lower than those in the parenteral nutrition group at the same time point (*P* < 0.05). At 3, 12, 24, and 48 hours after the operation, the levels of PvO_2_ and ScvO_2_ in two groups were higher than those before treatment, and the enteral nutrition group was higher than the parenteral nutrition group at the same time point (*P* < 0.05). After treatment, the levels of HGB, ALB, and TP in two groups were higher than those before treatment, and the enteral nutrition group was higher than the parenteral nutrition group (*P* < 0.05). After treatment, the nutritional scores of the two groups were higher than those before treatment, and the enteral nutrition group was higher than the parenteral nutrition group (*P* < 0.05). At 6-month postoperative follow-up, the incidence of death in the enteral nutrition group 2.44% (1/41) was lower than that of the parenteral nutrition group 17.07% (7/41) (*P* < 0.05).

**Conclusions:**

The efficacy of NIPPV combined with enteral nutrition support in treating patients with combined respiratory failure after lung cancer surgery is remarkable. It can improve patients' pulmonary function and blood gas index, correct patients' hypoxia status and the patients' nutritional level was significantly improved, which helped to reduce the mortality rate and improve the prognosis.

## 1. Introduction

Combined with the 2020 “Global Cancer Statistical Report,” in 2020, the number of cancer deaths in my country was about 3 million, of which nearly 715,000 were lung cancer, accounting for about 17.9% of the total number of new cancer cases in China, accounting for about 23.8% of cancer deaths, and its morbidity and mortality rank first among the new cases of malignant tumors [1]. In 2021, the number of new lung cancer cases in my country is about 783,700, and the number of deaths due to lung cancer was about 631,000. Its morbidity and mortality still rank first among malignant tumors [2]. Report [3] pointed out that lung cancer mortality associated with all risk factors increases with age, and with the intensification of population aging in my country, the proportion of lung cancer patients over 70 years old is increasing, so the treatment of lung cancer patients has attracted more and more attention. According to the recommendation of the National Comprehensive Cancer Network [4], surgery is the first choice for the treatment of early-stage lung cancer, especially for stage I-IIIA lung cancer. Clinically, more and more elderly lung cancer patients choose comprehensive treatment based on anatomical pneumonectomy. However, due to the poor physical fitness of elderly patients, they are often combined with chronic diseases of varying degrees, such as diabetes, asthma, chronic bronchitis, and emphysema, resulting in problems such as decreased cardiopulmonary function, poor stress and tolerance, and reduced resistance. For this reason, postoperative pulmonary complications (PPCs) occur more frequently, and respiratory failure is one of the most common PPCs in elderly lung cancer patients, which has a very poor prognosis and a high mortality rate. Therefore, targeted clinical preventive measures must be taken to reduce patient respiratory failure and improve prognostic survival. Ventilator-assisted ventilation as a form of positive pressure ventilation via nose and/or mask is now widely used in the treatment of various types of respiratory failure and has an overall efficiency rate of 51% to 91% [5]. But the effect of its use in patients with combined respiratory failure after lung cancer surgery has rarely been reported and is insufficient to form a valid argument.

In addition, since lung cancer is a malignant wasting disease, with the extension of the disease, the patient's body may have different degrees of nutritional disorders. This is coupled with the fact that the patient's body function decreases with age and lacks the ability to recover from the disease, which increases the occurrence of malnutrition, which is not only detrimental to the recovery of various physiological indicators and physical functions of the patient but also increases the incidence of complications and affects their prognosis. Some studies [6,7] have shown that enteral nutrition support can improve and maintain the immunity and metabolism of the organism effectively by providing nutritional substrates required for cellular metabolism, which therefore has the effect of enhancing the resistance of the organism and promoting disease recovery. This paper discusses the effect of noninvasive positive pressure ventilation (NIPPV) combined with enteral nutrition support in the treatment of patients with combined respiratory failure after lung cancer surgery and its effect on patients' blood gas indexes. Details are as follows.

## 2. Materials and Methods

### 2.1. General Information

From March 2016 to September 2021, 82 patients with combined respiratory failure after lung cancer surgery who were treated in our hospital were selected as the research subjects, including 52 males and 30 females, aged 60–80 years old, with an average age of 69.79 ± 3.18 years old. Inclusion criteria included the following: all patients had completed lung tumor resection and had complete postoperative pathology reports; clinical stage of lung cancer was stage I-III; diagnostic criteria for type I respiratory failure (blood oxygen partial pressure (PaO_2_) < 60 mmHg and partial pressure of carbon dioxide (PaCO_2_) was normal when the patient inhaled air at rest) and type II respiratory failure (PaO_2_ < 60 mmHg and PaCO_2_ > 50 mmHg when the patient inhaled air at rest) were met; expected postoperative survival time ≥6 months; postoperative hemodynamic stability; postoperative consciousness and consent to ventilator-assisted ventilation; ability to cough and cough up sputum and other airway protection; those with complete and compliant medical records; those who were informed and signed the consent form for this study. Exclusion criteria included the following: those with more airway secretions and sputum disturbance affecting ventilation; upper gastrointestinal bleeding and severe hypoxemia (PaO_2_ <45 mmHg); postoperative confusion or mental illness; combined autoimmune disease; combined other organ or system failure; respiratory failure secondary to other organ or system failure; previous facial and neck trauma, burns, and surgical history. All patients were equally divided according to the random number table method into the parenteral nutrition group (*n* = 41) treated with NIPPV + parenteral nutritional support and the enteral nutrition group (*n* = 41) treated with NIPPV + enteral nutritional support. The general data of the two groups of patients are shown in Table 1, which were not statistically significant and were comparable (*P* < 0.05).

### 2.2. Methods

Both groups were routinely given intravenous pain pumps for continuous postoperative pain relief, antibiotics and expectorant cough suppressants, nebulized inhalation, back patting therapy, etc. Vital signs were closely monitored during the period.

#### 2.2.1. Parenteral Nutrition Group Received NIPPV + Parenteral Nutrition Support Treatment

NIPPV operation: the patient was supine at 30–45°, and the VENTImotion 30 noninvasive ventilator (Weinmann, Germany) was used for treatment. The S-T breathing mode was adjusted according to the patient's specific conditions, and the ventilator parameters were set to respiratory rate <30 breaths/min, respiratory tidal volume >7 ml/kg, PaO_2_ at 60∼90 mmHg, PaCO_2_ at 40∼50 mmHg (1 mmHg = 0.133 kPa), and oxygen concentration was set at 90%–95% oxygen saturation. The ventilator parameters were adjusted according to the changes in the condition to ensure stable breathing and smooth airway, avoid respiratory fatigue, and gradually extend the duration of offline when the patient is in remission. Parenteral nutrition support: the average daily basal energy expenditure (BEE) was estimated according to the Harris-Benedict formula, among them, male BEE = 66.5 + 13.7 × weight (kg) + 5.0 × height (cm)−6.8 × age (y), female BEE = 65.1 + 9.5 × weight (kg) + 1.8 × height (cm)−4.7 × age (*y*). On this basis, the correction factor was adjusted according to the patient's fever and respiratory failure. The average daily nitrogen intake was 0.15∼0.2 g/kg, and the nutrition mixture was infused by deep venous drip for 2 weeks.

#### 2.2.2. Enteral Nutrition Group Received NIPPV + Enteral Nutrition Support Treatment

The NIPPV operation was the same as that of the parenteral nutrition group. Enteral nutrition support: a nasogastric tube was placed and whole protein enteral nutrition was infused with an initial amount of 750 kcal/d at 38°C via a nutrition pump at a controlled rate of 70–150 ml/h. Calories were gradually increased to a predicted value, predicted value = BEE × 1. 1× activity coefficient × correction factor C (male/female: 1. 16/1. 19), held for 2 weeks.

### 2.3. Observation Indicators

#### 2.3.1. Efficacy Assessment: The Total Effective Number Is the Sum of the Significantly Effective and Effective Numbers

Significantly effective: after treatment, PaO_2_ increased by >5%, oxygen saturation by >90%, the heart rate and respiratory rate improved significantly. Effective: after treatment, the respiratory rate improved significantly, but PaO_2_ and oxygen saturation did not. Ineffective: after treatment, PaO_2_, oxygen saturation, and the respiratory rate did not change.

#### 2.3.2. Pulmonary Function Indexes

The maximum expiratory pressure (PEmax), maximum midexpiratory flow rate (MMF), and maximum ventilation volume (MVV) were measured before and 3, 12, 24, and 48 h after treatment in both groups. The detection instrument was a CHEST-HI-701 type lung function tester (CHEST, Japan).

#### 2.3.3. Blood Gas Indexes

PaO_2_ and PaCO_2_ were measured before and 3, 12, 24, and 48 h after treatment in both groups. The detection instrument was a Cobas b123 blood gas analyzer (Roche, Germany).

#### 2.3.4. Oxygen Metabolism Indicators

The mixed venous oxygen tension (PvO_2_) and central venous oxygen saturation (ScvO_2_) were measured before and 3, 12, 24, and 48 h after treatment in both groups. The detection equipment was the same as the blood gas index.

#### 2.3.5. Nutritional Status Indicators

Hemoglobin (HGB), serum albumin (ALB), and total protein (TP) were detected before and after treatment in both groups. The detection instrument was the Beckman Coulter AU5800 automatic biochemical analyzer (Beckman Coulter Trading (China) Co., Ltd.).

#### 2.3.6. Nutritional Score

The Miniature Nutritional Assessment (MNA) method was implemented to assess the nutritional status of patients before and after the treatment, and the assessment items included 18 items such as overall assessment, dietary assessment, and anthropometric measurements, with a total score of 30. An MNA score of <17 indicated malnutrition, 17∼ < 24 indicated potential malnutrition, and ≥24 indicated good nutrition.

#### 2.3.7. Follow-up Situation

The two groups were followed up at 6 months after surgery for clinical symptoms (significant physical wasting, gastrointestinal bleeding, electrolyte disturbances, etc.) and death.

### 2.4. Statistical Methods

The SPSS 22.0 statistical software was used to process the data. Measurement data ($\bar{x}$ ± *s*) were compared between groups by the *t*-test, and enumeration data (%) were compared between groups by the *χ*^2^ test. *P* < 0.05 means the difference is statistically significant.

## 3. Results

### 3.1. Comparison of Efficacy Assessment between Two Groups

As shown in Figure 1, after treatment, the total effective rate of the enteral nutrition group 95.12% (39/41) was higher than that of the parenteral nutrition group 80.49% (33/41) (*P* < 0.05).

### 3.2. Comparison of Pulmonary Function Indexes between Two Groups

As shown in Figure 2, at 3, 12, 24, and 48 hours after the operation, the levels of PEmax, MMF, and MVV in two groups were higher than those before treatment, and the enteral nutrition group was higher than the parenteral nutrition group at the same time point (*P* < 0.05).

### 3.3. Comparison of Blood Gas Indexes between Two Groups

As shown in Figure 3, at 3, 12, 24, and 48 hours after the operation, the PaO_2_ levels in two groups were higher than those before treatment, and the PaCO_2_ levels were lower than those before treatment. The PaO_2_ levels in the enteral nutrition group were higher than those in the parenteral nutrition group at the same time point, and the PaCO_2_ levels were lower than those in the parenteral nutrition group at the same time point (*P* < 0.05).

### 3.4. Comparison of Oxygen Metabolism Indexes between Two Groups

As shown in Figure 4, at 3, 12, 24, and 48 hours after the operation, the levels of PvO_2_ and ScvO_2_ in two groups were higher than those before treatment, and the enteral nutrition group was higher than the parenteral nutrition group at the same time point (*P* < 0.05).

### 3.5. Comparison of Nutritional Status between Two Groups

As shown in Figure 5, after treatment, the levels of HGB, ALB, and TP in two groups were higher than those before treatment, and the enteral nutrition group was higher than the parenteral nutrition group (*P* < 0.05).

### 3.6. Comparison of Nutritional Scores between Two Groups

As shown in Figure 6, after treatment, the nutritional scores of two groups were higher than those before treatment, and the enteral nutrition group was higher than the parenteral nutrition group (*P* < 0.05).

### 3.7. Comparison of Follow-Up Situations between Two Groups

As shown in Figure 7, at 6-month postoperative follow-up, the incidence of death in the enteral nutrition group 2.44% (1/41) was lower than that of the parenteral nutrition group 17.07% (7/41) (*P* < 0.05).

## 4. Discussion

In addition to pneumonia, atelectasis, acute exacerbation of interstitial pneumonia, acute lung injury, pulmonary embolism, multiple lung cancer, and other intrapulmonary factors, the causes of respiratory failure after lung cancer surgery also include extrapulmonary factors such as liver dysfunction, ischemic heart disease, and central nervous system disorders; patient factors such as preoperative hypoxemia, smoking index, body mass index, anesthesia time; and surgical factors such as anesthesia time, thoracotomy time, and operation time [8–11]. From the above, it can be seen that the lung function damage caused by whatever reason can be regarded as the initiating factor of postoperative respiratory failure, and conventional oxygen therapy, bronchodilators, and other respiratory medical treatments cannot effectively reverse the lung function damage. In addition, affected by the poor body status and immune function of lung cancer patients, the patients eventually develop respiratory failure. Based on the above, there is an urgent clinical need to strengthen the intervention of respiratory failure after lung cancer resection to help patients smoothly pass the postoperative dangerous period, reduce the mortality rate, and improve their prognosis.

The efficacy of NIPPV in the treatment of severe respiratory failure has been clinically recognized [12,13]. Its mechanism of action is mainly to re-expand atrophied alveoli through effective ventilation, to improve respiratory muscle function, and reduce oxygen consumption, thereby correcting hypercapnia. It also removes respiratory secretions, reduces airway obstruction, improves oxygenation function, overcomes endogenous positive endocardial respiratory pressure, and improves respiratory muscle fatigue, thus relieving the symptoms of respiratory failure; and reduces the magnitude of negative thoracic pressure fluctuations to stabilize patient hemodynamics [14]. At the same time, NIPPV increases lung compliance and lung volume, minimizes further deterioration, reduces the probability of tracheal intubation, and reduces organism traumatization [15]. However, in view of the fact that the NIPPV cannot be removed from the mask in the early stage and the symptoms of dry throat are prone to occur, the patient's eating status is affected. To make up for this deficiency, patients need to be given adequate nutritional support in clinical practice. In this study, we applied NIPPV combined with nutritional support therapy to patients with complicated respiratory failure after lung cancer surgery and compared the effectiveness of combined parenteral nutritional support or enteral nutritional support therapy on top of NIPPV and the effects on various indexes of patients.

In this result, the total effective rate of the enteral nutrition group was higher than that of the parenteral nutrition group at 3, 12, 24, and 48 hours after the operation. The levels of PEmax, MMF, MVV, PaO_2_, PvO_2_, and ScvO_2_ in the two groups were higher than those before treatment, the PaCO_2_ levels were lower than those before treatment, and the levels of the above indicators in the enteral nutrition group were significantly improved compared with those in the parenteral nutrition group. It is suggested that compared with NIPPV + parenteral nutrition support treatment, NIPPV + enteral nutrition support treatment has a significant effect and can more quickly improve the lung function and blood gas indicators and correct the hypoxic state of elderly patients with lung cancer after surgery complicated with respiratory failure, which can create favorable conditions for active postoperative treatment. The reason may be related to the following two aspects: ① NIPPV connects the patient to the ventilator through a nasal and/or mask connection to provide positive pressure ventilation, which can provide airway-assisted ventilation and increase lung volume, etc. This method of ventilation has led to significant improvements in ventilator-assisted ventilation technology, such as ventilation mode, human-machine synchronization, nasal and/or mask sealing, comfort, and dead space reduction [16,17]. As for patients with combined respiratory failure after lung cancer surgery, the application of NIPPV can increase ventilation, promote lung reopening, reduce lung function impairment, improve gas distribution in the lesion area, and thus increase effective alveolar ventilation, while NIPPV has the effect of correcting hypoxia and carbon dioxide retention by improving gas distribution and the ventilation to blood flow ratio [18]. ② The application of enteral nutritional support, which delivers nutritional preparations into the digestive system through a nasal cannula, is more in line with human physiology than parenteral nutrition. Nutrients stimulate gastrointestinal peristalsis. The application of enteral nutrition can avoid the atrophy of the gastrointestinal mucosa and at the same time ensure the balance of the gastrointestinal flora, it also reduces the incidence of intestinal infection [19]. Moreover, enteral nutrition can improve the abnormalities of gastrointestinal function caused by hypoxia and hypercapnia, so it is beneficial to improve the absorption of nutrients in the body [20]. Additionally, enteral nutrition is convenient and inexpensive to administer, and for lung cancer patients, it can reduce their psychological guilt, resulting in higher patient acceptance and better compliance.

In the present results, after treatment, the HGB, ALB, TP levels and nutritional scores in two groups were higher than those before treatment, and the enteral nutrition group was higher than the parenteral nutrition group. At 6-month postoperative follow-up, the death rate occurred in the enteral nutrition group was lower than that in the parenteral nutrition group. This indicated that compared with NIPPV + parenteral nutrition support, NIPPV + enteral nutrition support was more helpful in improving the nutritional status and survival rate of elderly patients with combined respiratory failure after lung cancer surgery. The development of nutritional support therapy can improve and maintain the function and metabolism of the patient's cells and organisms, which has a positive significance for the recovery of the patient's physical function. And enteral nutrition is a new nutritional method, which is administered during surgery with tube placement, which not only has the advantage of being non-invasive, but also reduces complications such as hyperthermia, bleeding, and hemothorax; In addition, compared with intravenous nutrition supported by parenteral nutrition, the application of this therapy is mainly absorbed through the portal vein system, which can play the function of the body's organs to mediate normal nutrients to promote the recovery of gastrointestinal digestion and absorption capacity, and the patient's HGB, ALB, and TP levels rise, which not only has an important role in enhancing the immune function and nutritional status of patients with combined respiratory failure after lung cancer surgery but also leads to a reduction in the incidence of nosocomial infections such as pulmonary infections [21,22]. All of the above can create favorable conditions for the postoperative survival of patients, so the patients in the enteral nutrition group have a lower mortality rate, and the effect of improving respiratory failure is more significant and rapid.

In short, the efficacy of NIPPV combined with enteral nutrition support in treating patients with combined respiratory failure after lung cancer surgery is remarkable, which can improve patients' pulmonary function and blood gas index, correct patients' hypoxia status, and the patients' nutritional level was significantly improved, which helped to reduce the mortality rate and improve the prognosis.

## Figures and Tables

**Figure 1:** Comparison of efficacy assessment between the two groups. (a) Cases of efficacy assessments. (b) Percentage of efficacy assessments. ^*∗*^There was a statistical difference between two groups.

**Figure 2:** Comparison of pulmonary function indexes between two groups. (a) Pemax level. (b) MMF levels. (c) MVV levels. ^*∗*^Comparison with the same group before treatment, ^#^comparison with the parenteral nutrition group at the same time point. There is a statistical difference.

**Figure 3:** Comparison of blood gas indexes between two groups. (a) PaO_2_ level. (b) PaCO_2_ level. ^*∗*^Comparison with the same group before treatment, ^#^comparison with the parenteral nutrition group at the same time point. There is a statistical difference.

**Figure 4:** Comparison of oxygen metabolism indexes between two groups. (a) PvO_2_. (b) ScvO_2_. ^*∗*^Comparison with the same group before treatment, ^#^comparison with the parenteral nutrition group at the same time point. There is a statistical difference.

**Figure 5:** Comparison of nutritional status between two groups. (a) HGB level. (b) ALB level. (c) TP level. ^*∗*^Comparison with the same group before treatment, ^#^comparison with the parenteral nutrition group at the same time point. There is a statistical difference.

**Figure 6:** Comparison of nutritional scores between the two groups. ^*∗*^Comparison with the same group before treatment, ^#^comparison with the parenteral nutrition group after treatment. There is a statistical difference.

**Figure 7:** Comparison of follow-up situations between two groups. (a) Case of follow-up situation. (b) Percentage of follow-up situation. ^*∗*^There was a statistical difference between two groups.

**Table 1:** Comparison of general data between two groups.

	Parenteral nutrition group (*n* = 41)	Enteral nutrition group (*n* = 41)	*t*/*χ*^2^	*P*
Age (years old)	69.20 ± 3.20	70.39 ± 3.09	1.713	0.091
Male/Female (case)	25/16	27/14	0.210	0.647
Smoking history (n, %)	11 (26.83)	8 (19.51)	0.617	0.432
COPD history (*n*, %)	14 (34.14)	15 (36.59)	0.053	0.817
Lung cancer types (*n*, %)			0.878	0.831
Adenocarcinoma	16 (39.02)	20 (48.78)		
Squamous carcinoma	17 (41.46)	14 (34.14)		
Adenosquamous carcinoma	4 (9.76)	4 (9.76)		
Small cell carcinoma	4 (9.76)	3 (7.32)		

## Data Availability

The data that support the findings of this study are available from the associated author upon reasonable request.
